# Stochastic Inventory Model for Minimizing Blood Shortage and Outdating in a Blood Supply Chain under Supply and Demand Uncertainty

**DOI:** 10.1155/2020/8881751

**Published:** 2020-08-29

**Authors:** Han Shih, Suchithra Rajendran

**Affiliations:** ^1^Department of Industrial and Manufacturing Systems Engineering, University of Missouri Columbia, Columbia, MO 65211, USA; ^2^Department of Marketing, University of Missouri Columbia, Columbia, MO 65211, USA

## Abstract

**Purpose:**

Blood, like fresh produce, is a perishable element, with platelets having a limited lifetime of five days and red blood cells lasting 42 days. To manage the blood supply chain more effectively under demand and supply uncertainty, it is of considerable importance to developing a practical blood supply chain model. This paper proposed an essential blood supply chain model under demand and supply uncertainty.

**Methods:**

This study focused on how to manage the blood supply chain under demand and supply uncertainty effectively. A stochastic mixed-integer linear programming (MILP) model for the blood supply chain is proposed. Furthermore, this study conducted a sensitivity analysis to examine the impacts of the coefficient of demand and supply variation and the cost parameters on the average total cost and the performance measures (units of shortage, outdated units, inventory holding units, and purchased units) for both the blood center and hospitals.

**Results:**

Based on the results, the hospitals and the blood center can choose the optimal ordering policy that works best for them. From the results, we observed that when the coefficient of demand and supply variation is increased, the expected supply chain cost increased with more outdating units, shortages units, and holding units due to the impacts of supply and demand fluctuation. Variation in the inventory holding and expiration costs has an insignificant effect on the total cost.

**Conclusions:**

The model developed in this paper can assist managers and pathologists at the blood donation centers and hospitals to determine the most efficient inventory policy with a minimum cost based on the uncertainty of blood supply and demand. The model also performs as a decision support system to help health care professionals manage and control blood inventory more effectively under blood supply and demand uncertainty, thus reducing shortage of blood and expired wastage of blood.

## 1. Introduction

Blood and its components are all required in a variety of treatments, including cancer treatments, organ transplants, primary surgical operations, and trauma care. Even though substantial research has led to alternatives for blood, these endeavors have not been very fruitful so far. In 2013, it was reported that in the United States, there are around 15.2 million blood donors, and roughly 14.2 million units of blood were gathered, out of which, 13.2 million units were transfused [1].

The blood supply chain involves three main sectors: the hospitals—where the blood transfusion is ordered for patients, the blood center—a centralized location that receives requests from the hospitals, and the suppliers (blood donation sites)—an entity that is involved in donor management [2, 3]. The uncertainties in donations and demand for blood, the perishability of blood products, and the different echelons of the blood supply chain are the attributes and factors that have a substantial impact on the management of blood.

An interconnected series of blood management is called the blood supply chain management (BSCM). The significant challenges it faces are related to blood shortage, outdating, and supply chain costs, which are all needed to be minimized. An effective BSCM should be capable of handling blood demand while reducing shortage costs and wastage costs. Blood demand is highly liable to variation and attributes to scenarios with uncertainty. At the same time, the blood supply is also subject to significant uncertainty. The four main stages within BSCM include blood collection, production, inventory, and distribution of blood [4]. The level of effectiveness from the previous stage of the model will affect the following echelons in the blood supply chain. Previous researchers also considered health-related risks, supply readiness, fluctuation in demand, and short blood shelf life to the cost incurred during the entire process. Moreover, the uncertainty in blood supply and demand creates even more significant challenges for blood supply chain management.

Minimizing blood wastage and shortages poses a significant challenge in blood management at hospitals and blood centers [5]. On account of demand and supply uncertainty, mitigation efforts to manage and minimize the impact of outdated blood and shortages continue representing a challenging problem for hospitals [6]. Solyal et al. [7], Fortsch and Khapalova [8], and Rajendran and Ravindran [9] are the latest researchers who address the challenge in the inventory management of demand uncertainty. This paper extends the work by Rajendran and Ravindran [9] by developing a basic mathematical model under both blood supply and demand uncertainty.

This study focused on how to manage the blood supply chain under demand and supply uncertainty effectively. A stochastic mixed-integer linear programming (MILP) model for the blood supply chain is proposed incorporating the uncertain nature of both demand and supply. Furthermore, this study conducted a sensitivity analysis to examine the impacts of the coefficient of demand and supply variation (CV) and the cost parameters (CS) on the average total cost and the performance measures (units of shortage, outdated units, inventory holding units, and purchased units) for both the blood center and hospitals.

The remainder of the paper is organized as follows.  Section 2 presents the literature review. The finite-time horizon inventory blood supply chain model is discussed in Section 3, while the results and conclusions are, respectively, shown in Sections 4 and 5.

## 2. Literature Review

Research on optimizing and improving the efficiency of service systems, such as logistics, hospitality, health care, and education, has gained considerable attention in recent years (e.g., [10–15]). In particular, blood inventory management has attracted significant enthusiasm from the operation research scholars [16]. By far, the majority of the prior research has concentrated on the development of complex inventory models within the blood supply chain management. However, the advanced models proposed in the literature do not seem to be applied in practice [17]. Production does not take into consideration the critical age effect of inventory items [18]. Though there has been considerable research on blood inventory management related to the blood supply chain, the more substantial part of the literature focuses on one single echelon, and it does not examine the relationships among the different stages. As a result, it could cause a nearsighted perspective of the blood supply chain.

Gunpinar and Centeno [19] introduced a stochastic integer programming model within a planning horizon to reduce the shortage and wastage levels of blood components at a hospital. The models especially consider blood, considering the age of the blood unit for units stored in stock, the demands for two types of patients, the uncertainty in the demand rate, and the ratio of crossmatch to transfusion. Attari et al. [20] developed a goal programming model intending to diminish wastes and shortages of blood components in hospitals. These are all the instances of considering only a single echelon; however, the modeling of the complete process operation flow within the blood supply chain is particularly needed. Dillon et al. [21] suggested a two-stage stochastic programming model for determining superior policies for a periodic review of RBC inventory management in a blood supply chain. The model's goal is to reduce operating costs, blood shortages, and outdating as much as possible while considering the perishability and demand uncertainty.

Inventory management issues are significantly complicated by unknown demand [22]. Solyal et al. [7], Fortsch and Khapalova [8], and Rajendran and Ravindran [18] are some recent researchers who address demand uncertainty issues in inventory management. However, the inventory management taking the uncertainty attributes of demand and supply into account for the blood supply chain is needed to be studied. Blood supply chain management requires that both hospitals and blood centers are increasingly innovative and cost effective in collecting, producing, and delivering blood products and services [23–25]. It should take an appropriate approach to deal with inventory costs, blood platelet ages, the short shelf life of blood platelets, and also consider the demand and supply uncertainties.

### 2.1. Contributions to the Literature

We contribute to the current platelet inventory management literature multiple-folds. First, several blood inventory models proposed in the literature do not incorporate real-life constraints, such as demand uncertainty [9]. Dillon et al. [21] also observed that most of the blood inventory papers assume the demand to be deterministic. Nevertheless, Haijema et al. [26] highlighted that nearly 50% of the demand uncertainty is experienced at medical centers. This paper considers platelet demand uncertainty, and also the impact of the demand fluctuation is studied in detail. Second, this research is one of the very few articles to focus on developing inventory models for the entire blood supply chain (i.e., both hospitals and blood centers), instead of considering a single-stage problem.

Third, in addition to considering blood demand uncertainty, supply uncertainty is also incorporated in the proposed blood inventory model. This can enable decision makers to propose better recommendations on blood collection strategies. Fourth, this paper is one of the first to consider two types of demand at the blood center. The first is the regular demand received from the hospitals, and the second is the emergency demand ordered by hospitals when hospitals experience a shortage. The latter category of demand has to be immediately supplied to the hospitals, and these constraints are incorporated in the model proposed in this study.

## 3. Finite-Time Horizon Inventory (FTHI) Blood Supply Chain Model

This section presents a finite-time horizon inventory (FTHI) model to identify the optimal order quantity and time to order platelets such that wastage and shortages are reduced. A model for mixed-integer linear programming (MILP) is formed, and the platelet supply and demand for the planning horizon is given as an input to the model.  Figure 1 presents a structure of the blood supply chain containing one blood center and a *K* number of hospitals. The regulations of the Health Insurance Portability and Accountability Act (HIPAA) ensure that each hospital can receive blood only from a designated blood center and cannot share or procure blood from other hospitals.

### 3.1. Model Assumptions

1. Lead time for the order processing is assumed to be negligible.
2. This model considers a single blood type.
3. The FIFO issuing policy is applied at the hospital. That is, the platelet units with a one-day shelf life are first used for the demand fulfillment and then two-day and followed by three-day shelf life.

### 3.2. Scenario-Based Approach

A scenario-based approach is commonly used in the health care literature to consider uncertainty [18, 19, 27]. Similarly, in this research, a scenario optimization technique is utilized to solve the stochastic programming models by examining many possible circumstances for the platelet demand and supply. This approach is based on a set of key constraints for acquiring solutions to stochastic optimization problems. In a given period, each scenario corresponds to a specific combination of supply and demand patterns. Based on this stochastic programming approach, the number of acquired units with the regular shipments will remain the same, and the number of acquired units through emergency shipments (i.e., at times of shortage) and inventory is varied based on the scenario.

### 3.3. Notations for the Model

Parameters (known data) for the model:

 
*l*: index of platelets' shelf life (*l* = 1, 2, 3).
 
*k*: index of hospital *k*.
 
*s*: index of demand scenario (demand patterns for platelets) (*s* = 1, 2,…, *S*).
 
*t*: index of day *t* (*t* = 1, 2,…, *T*).
 
*K*: total number of hospitals (*K* = 1, 2,…, *K*).
  pb(*s*): probability of scenario *s*(∑_1_^*s*^pb(*s*)=1).
  foH*P*_*k*_: fixed operating cost per day at the hospital *k* ($/day).
  fsH*P*_*k*_: fixed shipping cost of purchasing platelets at hospital *k* ($/shipment).
  pcH*P*_*k*_: platelet purchasing cost for each unit by hospital *k* ($).
  hcH*P*_*k*_: holding cost for each inventory unit of platelet per day at hospital *k* ($/day/unit).
  ecH*P*_*k*_: cost of outdated platelet for each unit at hospital *k* ($).
  scH*P*_*k*_: shortage cost for each unit at hospital *k* ($) (this is referring to the procurement cost for each unit of platelet incurred through emergency shipment from the blood center).
  DEMAND_*k*,*t*_(*s*): platelet demand at hospital *k* at day *t* (units) under scenario *s*. The demand pattern can be estimated from historical data.
  LTHP_*k*_: lead time (days) of procurement at hospital *k*. It is the time between issuing orders for the platelet and receiving the platelet (note: LTHP_*k*_ = 0, 1, or 2 only).
  RPHP_*k*_: order review period at hospital *k* (days).
  iniHP_*k*,*l*_: beginning inventory at the hospital *k* on day 1 with *l* days of shelf life.
  foBC: fixed operating cost per day incurred at the blood center ($/day).
  fsBC: fixed shipping cost per shipment of purchasing platelets associated with the blood center ($/shipment).
  pcBC: removal of platelet and testing cost for each unit associated with the blood center ($/unit).
  hcBC: inventory holding cost for each unit per day of platelet associated with the blood center ($/day).
  esBC: cost of the outdated platelet for each unit associated with the blood center ($/unit).
  scBC: shortage cost per unit ($/unit) associated with the blood center (this is referring to the procuring cost for each unit of platelet incurred through emergency shipment from other blood centers).
  SUPPLY_*t*_(*s*): platelet supply at the blood center (units) at day *t* under scenario *s*. The supply pattern can be estimated from historical data.
  LTBC: lead time (days) for blood center procurement of platelets. It is the time between issuing orders and receiving fresh new platelets. It includes the time for collecting blood and two days for the testing time.
  RPBC: the review period for platelets ordering at the blood center (days).
  iniBC_*l*_: beginning inventory at the blood center on day one with *l* days of shelf life.

### 3.4. Main Decision Variables in Association with the Model

  TCSC: expected total cost gathered across the finite time (*T*) period for all scenarios of the blood supply chain.
  ORHP_*k*,*t*_(*s*): at the end of day *t*, the number of platelet units ordered by hospital *k*, under scenario *s*.
  REHP_*k*,*t*_(s): at the start of day *t*, the number of units that hospital *k* obtained from the blood center with *l* days of shelf life (*l* = 1,2,3) from the blood center, under scenario *s* (note: the arriving platelets have the maximum shelf life of three days).
  OHHP_*k*,*t*,*l*_(*s*): at the start of day *t*, the readily available inventory of platelet with *l* days of shelf life (*l* = 1, 2) at hospital *k*, under scenario *s*. Note: since platelets possess a maximum shelf life of three days when they are delivered to the hospital, the inventory available at the start of day *t* (brought over from day *t*−1) can possess a maximum of two days of shelf life.
  SHHP_*k*,*t*_(*s*): at the end of day *t*, the shortage of platelet units at hospital *k*, under scenario *s* (note: these are procured units from the blood center through the request of emergency shipment by the hospital *k*).
  EXHP_*k*,*t*_(*s*): at the end of day *t*, the expired platelet units at the hospital *k*, under scenario *s*.

### 3.5. Main Decision Variables in Association with the Blood Center for the Model

  ORBC_*t*_(s): at the end of day *t*, platelet units procured by the blood drives under scenario *s*. The blood center will receive these ordered platelet units at the start of day *t* + LTBC.
  REBC_*t*_(*s*): at the start of day *t*, the total amount of platelet arriving from the component labs to the blood center upon the completion of the testing process, under scenario *s* (note that all units of platelet received by the blood center will be fresh new and possess a three-day shelf life).
  BCTHP_*k*,*t*,*l*_(*s*): on day *t*, units shipped to hospital *k* with the platelets with *l* days of shelf life (*l* = 1, 2, 3) from the blood center, under scenario *s*.
  OHBC_*t*,*l*_(*s*): at the start of day *t*, the on-hand units of platelet with *l* days of shelf life (*l* = 1, 2) at the blood center, under scenario *s*. Note: since platelet units possess a maximum shelf life of three days, at the start of day *t*, the on-hand inventory (brought over from day *t* − 1) can possess a maximum shelf life of two days.
  SHBC_*t*_(s): at the end of day *t*, the shortage of platelets at the blood center under scenario *s*.
  EXBC_*t*_(s): at the end of day *t*, the number of expired platelet units at the blood center under scenario *s*.

### 3.6. Stochastic Integer Linear Programming for the Blood Supply Chain

#### 3.6.1. Sequence of Events at the Hospital

Beginning with the inventory of platelets with shelf lives of one day and two days
Receiving units of platelets from the blood center with one-, two-, and three-day shelf lives
Receiving the demand for platelets
Fulfilling the platelet demand at the hospital in the following order:
    Platelets with one-day shelf life are used first
    If insufficient, the platelets with two-day shelf life are used next
    Finally, the platelets with three-day shelf life are used
At the end of the day, reviewing the inventory of platelets and placing orders for new platelets following the ordering policy.

#### 3.6.2. Sequence of Events at the Blood Center

Beginning with the inventory of platelets with shelf lives of one day and two days
Replenishing the stock with new platelets arriving from the component labs with a shelf life of three days
Receiving regular demand from all the hospitals
Fulfilling the hospital demands in the following platelet order:
    Delivering platelets to hospital *k* with one-day shelf life first, provided hospital *k*'s lead time is zero days
    Next, delivering platelets to hospital *k* with two-day shelf life (if necessary), provided hospital *k*'s lead time is zero or one day
    Finally, shipping platelets to hospital *k* with a three-day shelf life (if necessary)
Receiving the demand for emergency from all hospitals
    Delivering platelets to all hospitals placing emergency demand with a one-day shelf life first, followed by two-day and three-day shelf life platelets if necessary.
Reviewing the inventory of platelets at the end of the day and placing orders for new platelets following the ordering policy.

### 3.7. Blood Supply Chain Model Formulation

Objective function: the objective of this model is to minimize the incurred total cost over the entire blood supply chain. There are 11 cost components associated with the entire blood supply chain:

The cost associated with hospital *k* on day *t*:
    Fixed operating cost: foHP_*k*_ × *t*
    Fixed transportation cost: fsHP_*k*_ × binHP_*k*,*t*_(*s*)
    Variable purchasing cost: pcHP_*k*_ × ORHP_*k*,*t*_(*s*)
    Inventory holding cost: hcHP_*k*_ × (OHHP_*k*,*t*,*1*_(*s*) *+* OHHP_*k*,*t*,2_(*s*))
    Shortage cost: scHP_*k*_ × SHHP_*k*,*t*_(*s*)
    Expiration cost: ecHP_*k*_ × EXHP_*k*,*t*_(*s*)
The cost related to the blood center on day *t*:
    Fixed operating cost: foBC × *t*
    Fixed transportation cost: fcBC × binBC_*t*_(*s*)
    Inventory holding cost: hcBC × (OHBC_*t,*1_(*s*) + OHBC_*t,*2_(*s*))
    Shortage cost: scBC × SHBC_*t*_(*s*)
    Expiration cost: ecBC × EXBC_*t*_(*s*)

Note: since this processing and testing cost will be covered by the various procurement costs paid by the hospitals, the objective function does not consider the cost of processing and testing platelets acquired at the blood center. The blood supply chain model under demand and supply uncertainty is formulated as follows:

(1) $$\begin{array}{c} \text{Minimize TCSC}=\sum_{t=1}^{T}\left[\sum_{s=1}^{S}\left[\text{pb}\left(s\right)\times \left\{\begin{array}{c} \sum_{k=1}^{k}\left[{\text{foHP}}_{k}\times t+{\text{fsHP}}_{k}+{\text{binHP}}_{k,t}\left(s\right)+{\text{pcHP}}_{k}\times {\text{ORHP}}_{k,t}\left(s\right)+{\text{hcHP}}_{k}\left({\text{OHHP}}_{k,t,1}\left(s\right)+{\text{OHHP}}_{k,t,2}\left(s\right)\right)+{\text{scHP}}_{k}\times {\text{SHHP}}_{k,t}\left(s\right)+{\text{ecHP}}_{k}\times {\text{EXHP}}_{k,t}\left(s\right)\right]\\ +\text{foBC}\times t+t+\text{fsBC}\times {\text{binBC}}_{t}\left(s\right)+\text{hcBC}\times \left({\text{OHBC}}_{t,1}\left(w\right)+{\text{OHBC}}_{t,2}\left(s\right)\right)+\text{scBC}\times {\text{SHBC}}_{t}\left(s\right)+\text{ecBC}\times {\text{EXBC}}_{t}\left(s\right) \end{array}\right\}\right]\right], \end{array}$$

(2) $$\begin{array}{c} {\text{REHP}}_{k,t,l}\left(s\right)={\text{BCTHP}}_{k,t-LTHP_{k},l+LTHP_{k}}\left(s\right),\;\forall t>{\text{LTHP}}_{k}\text{ and }l+{\text{LTHP}}_{k}\leq 3, \end{array}$$

(3) $$\begin{array}{c} {\text{REHP}}_{k,t,l}\left(s\right)=\text{0,}\;\text{otherwise,} \end{array}$$

(4) $$\begin{array}{c} {\text{DEMAND}}_{k,t}\left(s\right)-{\text{OHHP}}_{k,t,1}\left(s\right)-{\text{REHP}}_{k,t,1}\left(s\right)={\text{RDHP}}_{k,t,1}\left(s\right)-{\text{LYHP}}_{k,t,1}\left(s\right),\;\forall k,t,s, \end{array}$$

(5) $$\begin{array}{c} {\text{RDHP}}_{k,t,l}\left(s\right)-{\text{OHHP}}_{k,t,2}\left(s\right)-{\text{REHP}}_{k,t,2}\left(s\right)={\text{RDHP}}_{k,t,2}\left(s\right)-{\text{LYHP}}_{k,t,2}\left(s\right),\;\forall k,t,s, \end{array}$$

(6) $$\begin{array}{c} {\text{RDHP}}_{k,t,2}\left(s\right)-{\text{REHP}}_{k,t,3}\left(s\right)={\text{RDHP}}_{k,t,3}\left(s\right)-{\text{LYHP}}_{k,t,3}\left(s\right),\;\forall k,t,s, \end{array}$$

(7) $$\begin{array}{c} {\text{EXHP}}_{k,t}\left(s\right)={\text{LYHP}}_{k,t,1}\left(s\right),\;\forall k,t,s, \end{array}$$

(8) $$\begin{array}{c} {\text{OHHP}}_{k,t+1,1}\left(s\right)={\text{LYHP}}_{k,t,2}\left(s\right),\;\forall k,t,s, \end{array}$$

(9) $$\begin{array}{c} {\text{OHHP}}_{k,t+1,2}\left(s\right)={\text{LYHP}}_{k,t,3}\left(s\right),\;\forall k,t,s, \end{array}$$

(10) $$\begin{array}{c} {\text{SHHP}}_{k,t}\left(s\right)={\text{RDHP}}_{k,t,3}\left(s\right),\;\forall k,t,s, \end{array}$$

(11) $$\begin{array}{c} {\text{OHHP}}_{k,1,l}\left(s\right)={\text{iniHP}}_{k,l},\;\forall k,l,s, \end{array}$$

(12) $$\begin{array}{c} {\text{ORHP}}_{k,t,l}\left(s\right)=0,\;\forall k,t\neq {\text{RPHP}}_{k},2{\text{RPHP}}_{k},\ldots ,l,s, \end{array}$$

(13) $$\begin{array}{c} {\text{ORBC}}_{t}\left(s\right)=0,\;\forall t\neq \text{RPBC},2\text{RPBC},\ldots ,s, \end{array}$$

(14) $$\begin{array}{c} {\text{REBC}}_{t}\left(s\right)={\text{ORBC}}_{t-\text{LTBC}}\left(s\right),\;\forall t>\text{LTBC},s, \end{array}$$

(15) $$\begin{array}{c} {\text{ORBC}}_{t}\left(s\right)={\text{SUPPLY}}_{t}\left(s\right),\;\forall t,s, \end{array}$$

(16) $$\begin{array}{c} \sum_{k}{\text{BCTHP}}_{k,t,1}\left(s\right)+{\text{LFRBC}}_{t,1}\left(s\right)={\text{OHBC}}_{t,1}\left(s\right),\;\forall t,s,{\text{LTHP}}_{k}=0, \end{array}$$

(17) $$\begin{array}{c} \sum_{k}{\text{BCTHP}}_{k,t,2}\left(s\right)+{\text{LFRBC}}_{t,2}\left(s\right)={\text{OHBC}}_{t,2}\left(s\right),\;\forall t,s,{\text{LTHP}}_{k}=0,1, \end{array}$$

(in general, ∑_*k*_BCTHP_*k*,*t*,*l*_(*s*)+LFRBC_*t*,*l*_(*s*)=OHBC_*t*,*l*_(*s*), ∀*t*, *s*,  and *l*=1,2, LTHP_*k*_ ≤ *l*),

(18) $$\begin{array}{c} \sum_{k}\text{HP}3_{k,t}\left(s\right)+{\text{LFRBC}}_{t,3}\left(s\right)={\text{REBC}}_{t}\left(s\right),\;\forall t,s,{\text{LTHP}}_{k}=0,1,2, \end{array}$$

(19) $$\begin{array}{c} {\text{BCTHP}}_{k,t,1}\left(s\right)+{\text{BCTHP}}_{k,t,2}\left(s\right)+\text{HP}3_{k,t}\left(s\right)+{\text{SHRBC}}_{k,t}\left(s\right)={\text{ORHP}}_{k,t}\left(s\right),\;\forall t,k,s, \end{array}$$

(20) $$\begin{array}{c} {\text{BCTHP}}_{k,t,3}\left(s\right)=\text{HP}3_{k,t}\left(s\right)+{\text{SHRBC}}_{k,t}\left(s\right),\;\forall t,k,s, \end{array}$$

(21) $$\begin{array}{c} \sum_{k}{\text{SHHP}}_{k,t}\left(s\right)-{\text{LFRBC}}_{t,1}\left(s\right)={\text{RSHBC}}_{t,1}\left(s\right)-{\text{LFEBC}}_{t,1}\left(s\right),\;\forall t,s, \end{array}$$

(22) $$\begin{array}{c} {\text{RSHBC}}_{t,1}\left(s\right)-{\text{LFRBC}}_{t,2}\left(s\right)={\text{RSHBC}}_{t,2}\left(s\right)-{\text{LFEBC}}_{t,2}\left(s\right),\;\forall t,s, \end{array}$$

(23) $$\begin{array}{c} {\text{RSHBC}}_{t,2}\left(s\right)-{\text{LFRBC}}_{t,3}\left(s\right)={\text{RSHBC}}_{t,3}\left(s\right)-{\text{LFEBC}}_{t,3}\left(s\right),\;\forall t,s, \end{array}$$

(24) $$\begin{array}{c} {\text{SHEBC}}_{t}\left(s\right)={\text{RSHBC}}_{t,3}\left(s\right),\;\forall t,s, \end{array}$$

(25) $$\begin{array}{c} {\text{EXBC}}_{t}\left(s\right)={\text{LFEBC}}_{t,1}\left(s\right),\;\forall t,s, \end{array}$$

(26) $$\begin{array}{c} {\text{OHBC}}_{t+1,1}\left(s\right)={\text{LFEBC}}_{t,2}\left(s\right),\;\forall t,s, \end{array}$$

(27) $$\begin{array}{c} {\text{OHBC}}_{t+1,2}\left(s\right)={\text{LFEBC}}_{t,3}\left(s\right),\;\forall t,s, \end{array}$$

(28) $$\begin{array}{c} {\text{TSHBC}}_{t}\left(s\right)=\sum_{k}{\text{SHRBC}}_{k,t}\left(s\right)+{\text{SHEBC}}_{t}\left(s\right),\;\forall t,s, \end{array}$$

(29) $$\begin{array}{c} {\text{OHBC}}_{1,l}\left(s\right)={\text{iniBC}}_{l},\;\forall l,s, \end{array}$$

(30) $$\begin{array}{c} {\text{REHP}}_{k,t,l}\left(1\right)={\text{REHP}}_{k,t,l}\left(2\right)=\cdots ={\text{REHP}}_{k,t,l}\left(s\right),\;\forall k,t,l,s, \end{array}$$

(31) $$\begin{array}{c} {\text{ORHP}}_{k,t,l}\left(1\right)={\text{ORHP}}_{k,t,l}\left(2\right)=\cdots ={\text{ORHP}}_{k,t,l}\left(s\right),\;\forall k,t,l,s, \end{array}$$

(32) $$\begin{array}{c} {\text{REHP}}_{k,t,1}\left(s\right)+{\text{REHP}}_{k,t,2}\left(s\right)+{\text{REHP}}_{k,t,3}\left(s\right)\leq M\times {\text{binHP}}_{k,t}\left(s\right),\;\forall k,t,s, \end{array}$$

(33) $$\begin{array}{c} {\text{REBC}}_{t}\left(s\right)\leq M\times {\text{binBC}}_{t}\left(s\right),\;\forall t,s, \end{array}$$

(34) $$\begin{array}{c} {\text{REHP}}_{k,t,l}\left(s\right),{\text{RDHP}}_{k,t,l}\left(s\right),{\text{LYHP}}_{k,t,l}\left(s\right),{\text{OHHP}}_{k,t,l}\left(s\right),{\text{SHHP}}_{k,t}\left(s\right),{\text{ORHP}}_{k,t,l}\left(s\right), \end{array}$$

(35) $$\begin{array}{c} {\text{binHP}}_{k,t}\left(s\right)=0\text{ or }1,\;\forall k,t,s, \end{array}$$

(36) $$\begin{array}{c} {\text{binBC}}_{t}\left(s\right)=0\text{ or }1,\;\forall t,s. \end{array}$$

- *Units of Platelet Obtained by the Hospitalkfrom the Blood Center*: constraint (2) states that the total units obtained from the blood center by the hospital *k* with a shelf life of *l* days (REHP_*k*,*t*,*l*_(*s*)) will be equivalent to the units delivered from the blood center on day *t* − LTHP_*k*_, with a shelf life of *l*+LTHP_*k*_ days (note: LTHP_*k*_ = 0, 1, or 2 days).
- *Uncertainty Demand-Inventory Balance at Hospitalkand Daytunder Scenarios*: constraint (4) states that at hospital *k*, if stochastic demand DEMAND_*k*,*t*_(*s*) is higher than the units of platelet with one-day shelf life (i.e., DEMAND_*k*,*t*_(*s*) > OHHP_*k*,*t*,1_(*s*)+REHP_*k*,*t*,1_(*s*)), then the remaining demand denoted by RDHP_*k*,*t*,1_(*s*) is equal toDEMAND_*k*,*t*_(*s*)−OHHP_*k*,*t*,1_(*s*) − REHP_*k*,*t*,1_(*s*), and the leftover inventory with one-day shelf life denoted by LYHP_*k*,*t*,1_(*s*) will be 0. On the other hand, if DEMAND_*k*,*t*_(*s*) ≤ OHHP_*k*,*t*,1_(*s*)+REHP_*k*,*t*,1_(*s*), then RDHP_*k*,*t*,1_(*s*)=0 and LYHP_*k*,*t*,1_(*s*)=OHHP_*k*,*t*,1_(*s*)+REHP_*k*,*t*,1_(*s*) − DEMAND_*k*,*t*_(*s*). Equation (4) is used to calculate RDHP_*k*,*t*,1_(*s*) and LYHP_*k*,*t*,1_(*s*):
- If RDHP_*k*,*t*,1_(*s*) is positive, then the platelet units with two-day shelf life first fulfill the leftover demand (i.e., OHHP_*k*,*t*,2_(*s*)+REHP_*k*,*t*,2_(*s*)). If RDHP_*k*,*t*,1_(*s*) > OHHP_*k*,*t*,2_(*s*)+REHP_*k*,*t*,2_(*s*), then the leftover demand, RDHP_*k*,*t*,2_(*s*), will be equal to RDHP_*k*,*t*,1_(*s*) − OHHP_*k*,*t*,2_(*s*) − REHP_*k*,*t*,2_(*s*), and the remaining inventory with a shelf life of two days LYHP_*k*,*t*,2_(*s*) will be 0. On the other hand, if RDHP_*k*,*t*,1_(*s*) ≤ OHHP_*k*,*t*,2_(*s*)+REHP_*k*,*t*,2_(*s*), then RDHP_*k*,*t*,2_(*s*) = 0, and the remaining platelets with two-day shelf life are given by LYHP_*k*,*t*,2_(*s*)=OHHP_*k*,*t*,2_(*s*)+REHP_*k*,*t*,2_(*s*) − RDHP_*k*,*t*,1_(*s*). Equation (5) is used to calculate RDHP_*k*,*t*,2_(*s*) and LYHP_*k*,*t*,2_(*s*).
- If RDHP_*k*,*t*,2_(*s*) is positive, then the fresh platelet units with three-day shelf life (i.e., REHP_*k*,*t*,3_(*s*)) first fulfill RDHP_*k*,*t*,2_(*s*). If RDHP_*k*,*t*,2_(*s*) > REHP_*k*,*t*,3_(*s*), then the remaining demand, RDHP_*k*,*t*,3_(*s*), will be equal to RDHP_*k*,*t*,2_(*s*) − REHP_*k*,*t*,3_(*s*), and the remaining inventory with three-day shelf life, LYHP_*k*,*t*,3_(*s*), will be 0. If RDHP_*k*,*t*,2_(*s*) ≤ REHP_*k*,*t*,3_(*s*), then RDHP_*k*,*t*,3_(*s*)=0, and the remaining platelets with two-day shelf life are given by LYHP_*k*,*t*,3_(*s*)=REHP_*k*,*t*,3_(*s*) − RDHP_*k*,*t*,2_(*s*). Equation (6) is used to calculate RDHP_*k*,*t*,3_(*s*) and LYHP_*k*,*t*,3_(*s*).
- These above-specified FIFO rules are established using equations (4)–(6).
- *Expired (Outdated) Platelet Units at the Hospital*: constraint (7) states that at the end of day *t*, hospital *k* discards the unused platelet units with a remaining shelf life of one day (LYHP_*k*,*t*,1_(*s*)) and is given by equation (7).
- *Updates of Inventory at the Hospital*: the inventory at hospital *j* is updated at the end of each day using equations (8) and (9). Note that the ending inventory is varied for each hospital based on the scenario.
- *Platelet Shortages at the Hospital*: equation (10) represents the platelet shortages at the end of day *t* (SHHP_*k*,*t*_(*s*)) which is the unfulfilled demand, RDHP_*k*,*t*,3_(*s*).
- *Initial Inventory of Platelets at the Hospital*: equation (11) represents the beginning inventory at each hospital *k* at time *t* = 1 under each scenario *s*.
- *Platelet Units Ordered at the Hospital*: equation (12) states that the hospital *k* can only order platelets at the time of the review periods (*t*=RPHP_*k*_, 2RPHP_*k*_,…) and cannot order platelets at the time of the other days.
- *Units of Platelet Ordered and Received by the Blood Center*: similar to Constraint (12), equation (13) states that the blood center can only order platelets at the time of the review periods (*t*=RPBC, 2RPBC,…) and cannot order platelets at the time of the other days. At the blood center, upon the completion of the procedure of testing, the total available units at the start of day *t* under scenario *s* (REBC_*t*_(*s*)) are computed using equations (14) and (15). It has to be equivalent to the ordered amount placed prior to the lead time (ORBC_*t*−LTBC_(*s*)). Equation (15) states that the blood center has a stochastic supply at the start of each day *t* under scenario *s*, and the supply amount is estimated from historical real supply data.
- *Fulfillment for the Regular Platelet Demand by the Blood Center*: constraints (16)–(18) state that the total units of platelet distributed to the hospital *k* with *l* days of shelf life on the day *t* (BCTHP_*k*,*t*,*l*_(*s*)) are set as decision variables (i.e., the model determines the fulfillment policy for hospital demand), and they depend on the lead time of the hospital *k*. If the lead time at hospital *k* is one day because of the expiration of platelets at the time of arrival at the medical center, then the platelet units with a one-day shelf life should not be delivered to hospital *k* from the blood center. Hence, if the lead time at hospital *k* is one day, then platelet units distributed by the blood center should have two- or three-day shelf life. This is assured by equations (17) and (18). Likewise, if the lead time is two days at hospital *k*, then only platelet units with three-day shelf life have to be delivered to the hospital as given in equation (18). However, if the lead time of hospital *j* is zero days, then the platelet units with a shelf life of any day can be shipped as given in equations (16)–(18). As a result of the regular demand requested by hospital *k*,   the platelet shortage encountered at the blood center (SHRBC_*k*,*t*_(*s*)) is computed using equation (19). As reviewed previously, this shortage units will be acquired from other blood centers and fulfilled to the blood center. Within the proposed model, it is presumed that the procured shortage units SHRBC_*k*,*t*_(*s*) will possess a three-day shelf life. Therefore, although computing the platelet units which are delivered to the hospital by the blood center with the three-day shelf life category (i.e., BCTHP_*k*,*t*,3_(*s*)), SHRBC_*k*,*t*_(*s*) should also be incorporated alongside HP3_*k*,*t*_(*s*) (where HP3_*k*,*t*_(*s*) is the platelet units with three-day shelf life from the available inventory delivered to hospital *k*) as given in equation (20).
- *Fulfillment for the Emergency Demand by the Blood Center*: constraints (21)–(23) state that the regular demand placed by hospital *k* (ORHP_*k*,*t*_(*s*)) must be satisfied with the blood center, and the additional emergency demand requested on the same day *t* by that hospital (SHHP_*k*,*t*_(*s*)) is also satisfied with the blood center. As indicated in Section 3.4 regarding the processing of daily events, upon the fulfillment of regular demand(i.e., ∑_*k*_SHHP_*k*,*t*_(*s*) will be fulfilled with ∑_*l*_LFRBC_*t*,*l*_(*s*)), the emergency demand will be fulfilled only with inventory that is remaining in equations (21)–(23) which are like equations for regular demand-inventory balance conditions previously discussed.
- Note that LFEBC_*t*,*l*_(*s*)(*l*=1,2,3) in constraints (21)–(23) represents the remaining inventory of platelet units, with one-day, two-day, and three-day shelf life, upon completing the emergency orders of hospitals, and RSHBC_*t*,*l*_(*s*)(*l*=1,2,3) is the remaining shortage to be fulfilled by platelets. As a result of the emergency platelet demands requested by all the hospitals, the total shortage of platelets at the blood center is obtained by using equation (24).
- *Expired (Outdated) Platelets at the Blood Center*: at the end of each day *t*,  the expired platelet units at the blood center are obtained by using equation (25).
- *Updates of Inventory at the Blood Center*: at the end of each day *t*, the inventory at the blood center is updated by using equations (26) and (27).
- *Platelet Shortages at the Blood Center*: the platelet shortages at the blood center on each day *t*,  under scenario *s*, give the total scarcity as a result of the regular platelet demand (∑_*k*_SHRBC_*k*,*t*_(*s*)) as well as the emergency demand (SHEBC_*t*_(*s*)) requested by all the hospitals, as portrayed in equation (28).
- *Initial Inventory of Platelets at the Blood Center*: equation (29) gives the beginning inventory levels at the blood center at time *t*  = 1 for each scenario *s*.
- *Received Units for HospitalkHave to be the Same under All Scenarios*: equation (30) states that the received units for hospital *k* have to be the same for all scenarios over the supply chain planning horizon.
- *Ordered Units for HospitalkHave Equal Amount under All Scenarios over the Planning Horizon*: equation (31) states that the ordered units for hospital *k* have an equal amount for all the scenarios over the planning horizon.
- *Total Platelet Units Received by All Hospitals Shipped from the Blood Center*: equation (32) gives the total platelet units with *l* days of shelf life being received by all hospitals, at the start of day *t*.
- *Total Platelet Units Delivered to the Blood Center from the Component Labs*: equation (33) gives the total platelet units delivered from the component labs to the blood center upon the completion of the testing procedure, at the start of day *t*, under scenario *s*.
- *Nonnegative Integer Constraints*: constraint (34) represent nonnegative integer constraints in the model. Constraints (35) and (36) correspond to nonnegativity binary constraints within the model.

## 4. Computational Results

The model of the stochastic blood supply chain is programmed and solved using Python software with Gurobi Optimizer v8.1. The problem was solved to optimality for one blood center and two hospitals with a planning horizon of 300 days and 100 scenarios. It had 2,040,006 variables (90,000 are binary) and 1,621,202 constraints. It took about five minutes processing 417,279 iterations to solve the problem. Sections 4.1 and 4.2 discuss the results of computing solutions and sensitivity analysis in detail.

### 4.1. Base Case Results

This section examines the effectiveness of the developed stochastic mixed-integer programming model.  Table 1 shows the base case parameter values, and these are obtained from the literature [9, 18, 28, 29] for a setting with two hospitals and one blood supply chain. The impact of these cost parameters on the performance measures is discussed in Section 4.2.2.  Table 2 shows the performance measures and overall average cost measures for the base model with a planning horizon of 300 days and 100 scenarios. It is evident that Hospital #2 experiences more shortage, which is primarily because of the limited shelf life of arriving platelets. In other words, since the lead time for Hospital #2 is two days, there is comparatively more shortage and outdating observed in this hospital. As a result of the increased number of units purchased by Hospital #1, there are more units held in inventory, resulting in less shortage.

### 4.2. Sensitivity Analysis

In this section, the impact of supply and demand parameters, as well as the cost settings, is varied to investigate their effects on performance measures, such as shortage, outdating, holding, units purchased, and total cost.

#### 4.2.1. Impact of Changes on Demand and Supply Parameters

Table 3 shows the changes in coefficients of variation (CV) of both the supply and demand. The CV is varied from 10% to 50%, in steps of 0.1 at a time. Figures 2–4 show the impacts on performance measures for Hospitals #1 and #2 and the blood center, respectively.  Table 4 shows the overall average cost measures for different coefficients of demand and supply variations. Clearly, we can see that outdated units, held in inventory, and shortage increase with the inflation in the CV. Unexpectedly, the total units purchased decrease with the rise in CV for both the hospitals. The average supply at the blood center remains almost the same across the different CV settings and is approximately equal to the mean.

#### 4.2.2. Impact of Changes on the Cost Settings

Table 5 shows the different cost settings used for this analysis (adapted from [9]). Setting CSET1 represents the base case. Settings CSET2–CSET9 are obtained by multiplying the different cost parameters by 0.5, whereas settings CSET10–CSET17 are obtained by multiplying the different cost parameters by 1.5. Tables 6–8 show the impacts on average cost measures by different cost settings for different members of the supply chain. It is evident that settings with shortage cost variations have the maximum deviation from the base case. The next most significant impact is observed for purchasing cost parameter alteration. This is expected because the shortage cost has the maximum impact on the total cost. Due to the limited units outdated, the effect of varying the outdating cost parameters results in an insignificant change in the total cost. A similar pattern is observed for holding cost variations, as well.

## 5. Conclusions

The blood supply chain is genuinely unique as the products are very important to health care and life. Human blood cannot be manufactured, and no substitute for it has yet been successfully developed. Generally, many factors must be considered within the blood supply chain system because blood inventory management is a complex and challenging system. The collected donor blood faces a significant outdating because of the short shelf life of blood products. Moreover, hospitals and blood centers encounter serious blood inventory problems due to the uncertainty in blood demand and supply. In this study, we develop a stochastic mixed-integer linear programming model for the blood supply chain.

The problem with one blood center and two hospitals for a planning horizon frame of 300 days and 100 scenarios was solved to optimality using Python software with Gurobi Optimizer v8.1. It had 2,040,006 variables (90,000 are binary) and 1,621,202 constraints. It took about five minutes processing 417,279 iterations to solve the MILP problem. The results indicate that all the measures increase with the increase in the CV. This is because, with the increase in CV, more units are purchased to minimize shortage, which in turn results in more units held in inventory and more units expiring. It is also evident that settings with shortage and purchasing cost variations have the maximum deviation from the base case, while an insignificant change in the total cost is observed for holding and outdating cost variation settings.

Even though more effort is required in the implementation of the mathematical model and the forecasts have to be updated periodically, the model will result in less wastage and shortage. In practice, the same order policy may not be used for all the 300 days of the planning horizon. Instead, a rolling horizon approach may be followed to implement the optimal solution. For example, even though the MILP model gives an optimal order policy for 300 days, only the first week of the optimal solution is implemented. At the end of the first week, the MILP model is returned for the next 300 days after updating the inventory and demand forecast. The new optimal policy will be used for the second week, and the process is repeated weekly. Since long-term forecasts may not be as good as short-term forecasts, a rolling horizon policy helps to update forecasts weekly and determine the best solution based on the revised forecasts.

## Figures and Tables

**Figure 1:** Structure of the supply chain containing one blood center and *K* hospitals.

**Figure 2:** Impact of CV on performance measures of Hospital 1.

**Figure 3:** Impact of CV on performance measures of Hospital 2.

**Figure 4:** Impact of CV on performance measures of the blood center.

**Table 1:** Input parameters for the base case setting.

Input parameter	Values		
Total days over time horizon	300		
Total number of scenarios	100		

Hospitals/blood center	Hospital 1	Hospital 2	Blood center

Lead time (days)	1	2	5
Review period (days)	1	1	1
Fixed cost of procurement per shipment	113	225	1125
Inventory holding cost per unit per day	130	130	108
Variable purchasing cost per unit ($)	650	650	538
Shortage cost per unit ($)	3250	3250	2690
Outdating cost per unit ($)	650	650	538
Platelet demand/supply distribution	*N* ~ (200,32)	*N* ~ (100,16)	*N* ~ (225,36)

**Table 2:** Average performance measures for the base case setting (*T*=300, *S* = 100).

Performance measure	Hospital 1	Hospital 2	Blood center
Unit shortage	14	23	41
Unit outdating	0	1	0
Unit holding	21	0	1
Unit purchased	186	78	225
Fixed cost	1.13	2.25	11.25
Demand/supply	*N*∼(200, 32)	*N*∼(100, 16)	*N*∼(225, 37)

Overall measures			

Average cost/per day/per scenario	Best	Worst	STD
4,068	3,800	4,264	84

**Table 3:** Coefficients of variation (CV) of supply and demand settings.

Setting	Hospital 1	Hospital 2	Blood center
CV1 (CV = 0.1)	*N* ~ (200,20)	*N* ~ (100,10)	*N* ~ (225,23)
CV1 (CV = 0.2)	*N* ~ (200,40)	*N* ~ (100,20)	*N* ~ (225,45)
CV1 (CV = 0.3)	*N* ~ (200,60)	*N* ~ (100,30)	*N* ~ (225,68)
CV1 (CV = 0.4)	*N* ~ (200,80)	*N* ~ (100,40)	*N* ~ (225,90)
CV1 (CV = 0.5)	*N* ~ (200,100)	*N* ~ (100,50)	*N* ~ (225,115)

**Table 4:** Impact of CV on the total supply chain cost.

Overall measures				
Settings	Average cost/per day/per scenario	Best	Worst	STD
CV = 0.1	3,953	3,830	4,059	48
CV = 0.2	4,177	3,879	4,436	93
CV = 0.3	4,557	4,306	4,857	116
CV = 0.4	5,040	4,713	5,455	155
CV = 0.5	5,543	5,039	5,975	185

**Table 5:** Different settings of the cost.

Cost settings	Blood center			Hospital					
	Inventory holding cost (unit/day)	Shortage cost (unit)	Outdated cost (unit)	Fixed cost (shipment)		Inventory holding cost (unit/day)	Purchasing cost (unit)	Shortage cost (unit)	Outdated cost (unit)
				H1	H2				
CSET1 (base)	108	2690	538	(113, 225)		130	650	3250	650
CSET2	54	2690	538	(113, 225)		130	650	3250	650
CSET3	108	1345	538	(113, 225)		130	650	3250	650
CSET4	108	2690	269	(113, 225)		130	650	3250	650
CSET5	108	2690	538	(57, 113)		130	650	3250	650
CSET6	108	2690	538	(113, 225)		65	650	3250	650
CSET7	108	2690	538	(113, 225)		130	325	3250	650
CSET8	108	2690	538	(113, 225)		130	650	1625	650
CSET9	108	2690	538	(113, 225)		130	650	3250	325
CSET10	162	2690	538	(113, 225)		130	650	3250	650
CSET11	108	4035	538	(113, 225)		130	650	3250	650
CSET12	108	2690	807	(113, 225)		130	650	3250	650
CSET13	108	2690	538	(170, 338)		130	650	3250	650
CSET14	108	2690	538	(113, 225)		195	650	3250	650
CSET15	108	2690	538	(113, 225)		130	975	3250	650
CSET16	108	2690	538	(113, 225)		130	650	4875	650
CSET17	108	2690	538	(113, 225)		130	650	3250	975

**Table 6:** Impacts of cost settings on Hospital 1.

Average cost measures					
	Unit shortage	Unit outdating	Unit holding	Unit purchased	Total cost
CSET1 (base)	14	0	21	186	1917
CSET2	14	0	20	186	1916
CSET3	5	1	46	196	1729
CSET4	14	0	20	186	1916
CSET5	14	0	21	186	1805
CSET6	12	0	27	188	1856
CSET7	11	0	28	189	1234
CSET8	48	0	1	152	1995
CSET9	14	0	20	186	1916
CSET10	14	0	20	186	1916
CSET11	28	0	6	171	2255
CSET12	14	0	20	186	1916
CSET13	14	0	20	186	2030
CSET14	16	0	16	184	1973
CSET15	18	0	13	182	2602
CSET16	5	1	50	198	1828
CSET17	14	0	20	186	1916

**Table 7:** Impacts of cost settings on Hospital 2.

Average cost measures					
	Unit shortage	Unit outdating	Unit holding	Unit purchased	Total cost
CSET1 (base)	23	1	0	78	1261
CSET2	23	1	0	78	1261
CSET3	10	4	0	93	955
CSET4	23	1	0	78	1261
CSET5	23	1	0	78	1261
CSET6	24	0	0	77	1280
CSET7	19	1	0	82	890
CSET8	40	0	0	60	1040
CSET9	23	1	0	78	1257
CSET10	23	1	0	77	1254
CSET11	35	0	0	65	1560
CSET12	23	1	0	78	1261
CSET13	23	1	0	78	1261
CSET14	23	1	0	78	1261
CSET15	28	0	0	73	1621
CSET16	11	3	0	92	1153
CSET17	23	0	0	77	1248

**Table 8:** Impacts of cost settings on the blood center.

Average cost measures				
Setting	Unit shortage	Unit outdating	Unit holding	Total cost
CSET1 (base)	41	0	1	1103
CSET2	41	0	1	1103
CSET3	65	0	0	874
CSET4	41	0	1	1103
CSET5	41	0	1	1103
CSET6	43	0	0	1156
CSET7	48	0	1	1292
CSET8	9	0	1	243
CSET9	42	0	1	1130
CSET10	41	0	0	1102
CSET11	21	0	1	848
CSET12	41	0	1	1103
CSET13	41	0	1	1103
CSET14	40	0	1	1077
CSET15	33	0	1	888
CSET16	63	0	0	1694
CSET17	41	0	1	1103

## Data Availability

The data are obtained from prior studies.
